The article "Bicomponent polymeric micelles for pH-controlled delivery of doxorubicin" was retracted in 2024. Reasons: unreliable results or conclusions; concerns about the data.

# Bicomponent polymeric micelles for pH-controlled delivery of doxorubicin

**DOI:** 10.1080/10717544.2020.1726526

**Published:** 2020-02-24

**Authors:** Chunyun Wang, Peilan Qi, Yan Lu, Lei Liu, Yanan Zhang, Qianli Sheng, Tianshun Wang, Mengying Zhang, Rui Wang, Shiyong Song

**Affiliations:** Institute of Pharmacy, School of Pharmacy, Henan University, Kaifeng, China

**Keywords:** Drug delivery, pH-responsive, micelle, boronate ester, cancer

## Abstract

Stimuli-responsive drug delivery systems (DDSs) are expected to realize site-specific drug release and kill cancer cells selectively. In this study, a pH-responsive micelle was designed utilizing the pH-sensitivity of borate bonds formed between dopamine and boronic acid. First, methyl (polyethylene glycol)-block-polycaprolactone (mPEG-PCL) was conjugated with 4-cyano-4-(thiobenzoylthio)pentanoic acid (CTP) to obtain a macroinitiator. Two different segments poly(dopamine methacrylamide) (PDMA) and poly(vinylphenylboronic acid) (PVBA) were then grafted to the end of mPEG-PCL. Two triblock copolymers, mPEG-PCL-PDMA and mPEG-PCL-PVBA, were then obtained by reversible addition–fragmentation transfer (RAFT) polymerization. These copolymers and their mixture self-assembled in aqueous solution to form micelles that were able to load hydrophobic anticancer drug doxorubicin (DOX). These two-component micelles were found to be pH-sensitive, in contrast to the one-component micelles. Furthermore, MTT studies showed that the micelles were almost nontoxic. The DOX-loaded micelles showed cytotoxicity equivalent to that of DOX at high concentration. *In vivo* antitumor experiments showed that this pH-sensitive polymeric micellar system had an enhanced therapeutic effect on tumors. These two-component boronate-based pH micelles are universally applicable to the delivery of anticancer drugs, showing great potential for cancer therapy.

## 1. Introduction

Stimuli-responsive drug delivery systems (DDSs) have been developed to improve the insolubility and stability of anticancer drugs, and achieve controllable drug release, resulting in a better tumor inhibition effect and fewer toxic and side effects (Fernandes Stefanello et al., 2014; Ouahab et al., 2014; Davoodi et al., 2016; Wang et al., 2017; Pan et al., 2019). The tumor area has a special biochemical and physicochemical microenvironment that is different to normal tissues, such as a high intracellular ATP concentration, excessive expression of various biological enzymes, and a low pH value (Ganta et al., 2008; Aluri et al., 2009; Felber et al., 2012; Alex et al., 2017), which is the basis for the design of stimuli-responsive drug carriers for encapsulation and controlled anticancer drug release.

pH-responsive systems have been frequently employed and approved as among the most efficient drug delivery strategies (Torchilin, 2014; Mu et al., 2019). The pH value of tumor tissue is often 0.5–1.0 units lower than that of normal tissue. The lower pH value of the tumor, together with the acidic environments in endosomes and lysosomes, can be used as signals to trigger rapid drug release, the level of cells within the effective of swallowing and organelles targeted (Wu et al., 2019). Notably, pH-sensitive nanocarriers, which are stable at physiological pH values, but are capable of being triggered to release their payloads under acidic conditions in target tumors, may lead to a significantly improved therapeutic effect and minimal negative side effects.

The article "Bicomponent polymeric micelles for pH-controlled delivery of doxorubicin" was retracted in 2024. Reasons: unreliable results or conclusions; concerns about the data.

In the past decade, boronic acid and its derivatives, which can rapidly react with compounds containing 1,2- or 1,3-diol structures to form environment-pH-responsive boronic ester bonds, have attracted extensive interest. By taking advantage of the acidic hydrolysis properties of borate ester bonds, boronic acid-based pH-responsive DDSs are expected to realize site-specific drug release and kill cancer cells selectively (Liu et al., 2005; Zhong et al., 2010; Bartelmess et al., 2014). Wang et al. (2015) synthesized a boric acid-functionalized polymer that could be combined with polyphenolic anticancer drug emodin to form a pH-responsive prodrug. This prodrug had a considerable drug encapsulation efficiency of up to 78% and rapidly released emodin in an acidic environment. The inhibitory effect of this prodrug on HepG2 hepatocellular carcinoma cells was significantly higher than that on Mc-3T3-e1 normal cells, indicating a specific tumor inhibition effect. Su et al. (2011) combined Bortezomib (BTZ) with dopamine-functionalized polyethylene glycol to prepare pH-responsive DDSs. These pH-responsive DDSs showed high drug conjugation and a BTZ substitution degree of up to 50%. Meanwhile, 30% BTZ release was observed in pH 7.4 phosphate-buffered saline (PBS) within 12 h, which was increased to 80% at pH 5.0. Furthermore, these DDSs specifically inhibited the proliferation of MDA-MB-231 breast cancer cells, with a therapeutic effect about 2.2-fold higher than that of non-pH-responsive DDSs. Therefore, boronic acid-based DDSs show great potential for applications as anticancer drug carriers owing to their ability to selectively deliver drugs to tumor cells (Chen et al., 2012; Ren et al., 2013; Hasegawa et al., 2015; van der Vlies et al., 2016). However, pH-responsive DDSs can only be applied to drugs bearing boronic acid or 1,2-diol groups (Jia et al., 2015; Liu et al., 2018), with systems for common drugs, such as doxorubicin and paclitaxel, seldom reported.

The article "Bicomponent polymeric micelles for pH-controlled delivery of doxorubicin" was retracted in 2024. Reasons: unreliable results or conclusions; concerns about the data.

The stability of a micellar DDS is critically important. The cargo-loaded micelles should keep their integrity during the circulation process. To this end, the stability of micelles could be improved by introducing additional components, which could strengthen the molecular interaction of the micelles (Peng et al., 2019). In this study, a pH-responsive bicomponent micellar DDS was developed based on borate bond linkages. Firstly, two triblock copolymers, mPEG-PCL-PDMA and mPEG-PCL-PVBA, were synthesized, bearing oligomeric dopamine and phenylboronic acid segments, respectively. A micellar system with pH-sensitive boronate linkages was then formed by self-assembly of the mixture of these two amphiphilic polymers. Hydrophobic drug doxorubicin was encapsulated into the micelles. This DDS was expected to show pH-responsive drug release behavior and an enhanced therapeutic effect on tumors.

## 2. Materials and methods

### 2.1. Materials

Methyl poly(ethylene glycol) (mPEG, Mn = 5000 Da) and stannous octanoate (Sn(Oct)2, 95%) were purchased from Sigma-Aldrich (St. Louis, MO, USA). mPEG was dried in a vacuum oven at 37 °C before use. ε-Caprolactone (ε-CL) was obtained from Aladdin (Shanghai, China) and distilled from CaH_2_ under reduced pressure before use. 4-Dimethylaminopyridine (DMAP, 98%), *N*,*N*′-dicyclohexylcarbodiimide (DCC, 98%), and dopamine hydrochloride were obtained from Shanghai Darui Fine Chemical Co., Ltd., and used as received. 4-Cyano-4-(thiobenzoylthio)pentanoic acid (CTP, 97%) was supplied by J&K Scientific (Beijing, China) and used as received. Doxorubicin hydrochloride (DOX-HCl, 98%) was obtained from Dalian Meilun Biology Technology Co., Ltd. (Dalian, China) and stored in a refrigerator below 20 °C prior to use. 3-(4,5-Dimethyl-2-thiazolyl)-2,5-diphenyl-2*H*-tetrazolium bromide (MTT, 98%) and 4′,6-diamidino-2-phenylindole (DAPI, 90%) were supplied by Sigma (Shanghai, China) and stored in a refrigerator below 4 °C prior to use. All other reagents and chemicals were used as received.

Human L02 normal hepatocytes, human liver cancer cell line HepG-2, and human breast cancer cell line MCF-7 were supplied by Shanghai Cell Bank of the Chinese Academy of Sciences (Shanghai, China) and cultured in a humidified atmosphere containing 5% CO_2_ at 37 °C. Female Swiss mice (6–8 weeks old, 20 ± 2 g) were provided by the Medical Experimental Animal Center, Henan Province (Zhengzhou, China). Animal experiments were performed strictly according to the principles of care and use of laboratory animals, and were approved by the Animal Experimentation Ethics Committee of Henan University.

The article "Bicomponent polymeric micelles for pH-controlled delivery of doxorubicin" was retracted in 2024. Reasons: unreliable results or conclusions; concerns about the data.

### 2.2. Synthesis of block copolymers

#### 2.2.1. Synthesis of block copolymer mPEG-PCL

mPEG-PCL was synthesized using Sn(Oct)_2_ as catalyst. Typically, mPEG (2.0 g) and ε-CL (2.2 g) were dissolved in a certain amount of anhydrous toluene. After placing under vacuum and then purging with nitrogen gas, Sn(Oct)_2_ (100 μl) was added and the reaction mixture was stirred for 24 h at 115 °C. Upon reaction completion, the polymerization mixture was rapidly cooled and dissolved in dichloromethane (15 ml). The polymer was precipitated in ice-cold diethyl ether and isolated by filtration three times to obtain mPEG-PCL as a white solid (90% yield (by weight), molecular weight: 10,000 Da). ^1^H NMR (400 MHz, CDCl_3_, ppm): δ 4.05 (t, 2H, –CH_2_CH_2_O–), 3.65 (s, 4H,CH_3_OCH_2_CH_2_O–), 2.30 (t, 2H, –OOCH_2_CH_2_–), 1.64 (m, 4H, –CH_2_CH_2_CH_2_CH_2_CH_2_O–), 1.38 (t, 2H, –CH_2_CH_2_CH_2_–).

#### 2.2.2. Synthesis of macroinitiator mPEG-PCL-CTP

mPEG-PCL (3.3 g), CTP (0.46 g), and DMAP (61 mg) were dissolved in anhydrous dichloromethane (35 ml). DCC (0.72 g) was then added and the mixture was allowed to react at room temperature for 72 h. Upon reaction completion, the reaction mixture was filtered to remove the precipitate. The filtrate was extracted with hydrochloric acid and sodium bicarbonate, and then precipitated in ice-cold diethyl ether. The precipitate was isolated by filtration three times and then dried at 40 °C under vacuum. mPEG-PCL-CTP was obtained as a pink solid in 47.1% yield. ^1^H NMR (400 MHz, CDCl_3_, ppm): δ 7.91 (d, 2H, Ar-H), 7.56 (dd, 1H, Ar-H), 7.40 (t, 2H, Ar-H), 4.05 (t, 2H, –CH_2_CH_2_O–), 3.65 (s, 4H, CH_3_OCH_2_CH_2_O–), 2.30 (t, 2H, –OOCH_2_CH_2_–), 1.64 (m, 4H, –CH_2_CH_2_CH_2_CH_2_CH_2_O–), 1.38 (t, 2H, –CH_2_CH_2_CH_2_–).

#### 2.2.3. Preparation of monomer dopamine methacrylamide (DMA)

NaHCO_3_ (8.5 g) and Na_2_B_4_O_7_(H_2_O)_10_ (4.4 g) were dissolved in deionized water (100 ml). After placing under vacuum and then purging with nitrogen gas to create an anaerobic environment, dopamine–HCl (5.4 g) was added to the mixture, followed by dropwise addition of methacrylic anhydride (4.7 ml) in tetrahydrofuran (THF, 28 ml). The mixture was progressively adjusted to pH >8 by adding aqueous NaOH (1–5 M) and then stirred under nitrogen overnight. The reaction mixture was then adjusted to pH <2 by adding hydrochloric acid (6 M) and extracted four times with ethyl acetate (100 ml). The organic layer was dried over MgSO_4_ and concentrated by rotary evaporation. Hexane (100 ml) was added to the remaining residue for storage at –20 °C overnight to allow complete precipitation of the product. After drying at 50 °C under vacuum, DMA was obtained as a white solid in 89.3% yield (by weight). ^1^H NMR (400 MHz, d_6_-DMSO, ppm): δ 8.78 (1H, s, Ph-OH), 8.66 (1H, s, Ph-OH), 7.95 (1H, t, –CH_2_NHCO–), 6.64–6.41 (3 H, m, Ph), 5.62 (1H, s, CH_2_=C), 5.25 (1H, s, CH=C–), 3.22 (2H, q, –CH_2_CH_2_NH–), 2.5 (2H, tr, Ph–CH_2_CH_2_–), 1.8 (3 H, s, CH_3_C–).

The article "Bicomponent polymeric micelles for pH-controlled delivery of doxorubicin" was retracted in 2024. Reasons: unreliable results or conclusions; concerns about the data.

#### 2.2.4. Synthesis of amphipathic triblock copolymer mPE-PCL-PDMA

mPEG-PCL-PDMA was synthesized by reversible addition–fragmentation chain transfer (RAFT) polymerization. mPEG-PCL-CTP (0.65 g) was added to DMF (6 ml) and dissolved completely with sonication. After placing under vacuum for 25 min in an ice bath and then purging with nitrogen gas for 15 min, DMA (0.46 g) and AIBN (4 mg) were added, and the reaction mixture was stirred for 24 h at 75 °C. The reaction was stopped by rapidly cooling in an ice bath. The reaction mixture was diluted with DMF, transferred into a dialysis bag (molecular weight cutoff (MWCO), 8,000–14,000 Da), and dialyzed in distilled water for 24 h. The dialysis medium was refreshed every 6 h. Freeze-drying then afforded mPEG-PCL-PDMA as a powder in 87.8% yield (by weight) (molecular weight: 15,000 Da). ^1^H NMR (400 MHz, d_6_-DMSO, ppm): δ 8.78 (1H, s, Ph-OH), 8.66 (1H, s, Ph-OH), 7.40 (t, 2H, Ar-H), 6.64–6.41 (3 H, m, Ph), 4.05 (t, 2H, –CH_2_CH_2_O–), 3.65 (s, 4H, CH_3_OCH_2_CH_2_O–), 3.22 (2H, q, –CH_2_CH_2_NH–), 2.30 (t, 2H, –OOCH_2_CH_2_–), 1.64 (m, 4H, –CH_2_CH_2_CH_2_CH_2_CH_2_O–), 1.38 (t, 2H, –CH_2_CH_2_CH_2_–).

#### 2.2.5. Synthesis of amphipathic triblock copolymer mPEG-PCL-PVBA

mPEG-PCL-PVBA was synthesized using a similar to that of mPEG-PCL-PDMA, but with DMA replaced by 4-vinylphenylboronic acid (4-VBA), to obtain mPEG-PCL-PVBA as a sticky solid in 91.9% yield (by weight) (molecular weight: 15,000 Da). ^1^H NMR (400 MHz, d_6_-DMSO, ppm): δ 8.02–6.27 (m, aromatic protons), 4.05 (t, 2H, –CH_2_CH_2_O–), 3.65 (s, 4H, CH_3_OCH_2_CH_2_O–), 2.30 (t, 2H, –OOCH_2_CH_2_–), 1.64 (m, 4H, –CH_2_CH_2_CH_2_CH_2_CH_2_O–), 1.38 (t, 2H, –CH_2_CH_2_CH_2_–).

### 2.3. Characterization

^1^H NMR spectra of copolymers were recorded on a Bruker Fourier 400 NMR spectrometer in CDCl_3_ and d_6_-DMSO. Chemical shifts were calibrated against residual solvent signals. Fourier transformed-infrared spectroscopy (FTIR) was performed using an AVATAR360 (Nicolet, USA) spectrometer. The micelle size was determined by dynamic light scattering (DLS) at 25 °C using a Zetasizer Nano-ZS90 instrument (Malvern Instruments, UK) equipped with a 633-nm He–Ne laser. Morphological examinations were performed by transmission electron microscopy (TEM) (JEM-100CX II, JEOL, Tokyo, Japan) at an accelerating voltage of 100 kV. The molecular weight and polydispersity of the copolymers were determined by a Damn Eos (Wyatt, USA) gel permeation chromatograph (GPC) instrument equipped with Phenogel 10E6A column and a OPTILAB rEX refractive-index detector. Measurements were performed using tetrahydrofuran (THF) as the eluent at a flow rate of 1.0 mL/min at 30 °C and a series of narrow polystyrene standards for the calibration of the columns. All samples were obtained by filtering through a 0.22-μm Millipore filter into a clean scintillation vial.

The article "Bicomponent polymeric micelles for pH-controlled delivery of doxorubicin" was retracted in 2024. Reasons: unreliable results or conclusions; concerns about the data.

### 2.4. Micelle formation and pH-triggered changes in micelle size

The solvent evaporation method was used to prepare polymer micelles. First, mPEG-PCL-PDMA and mPEG-PCL-PVBA in a 1:1 molar ratio were dissolved in a mixture of THF and methanol, and the mixture was stirred at room temperature for 5 h. The mixture was then added dropwise into deionized water (30 ml, pH 8.5) under magnetic stirring at room temperature for 24 h. The resulting micelles were then filtered through a 0.22-μm syringe filter. The control group polymer micelles of mPEG-PCL-PDMA and mPEG-PCL-PVBA were similar to the mPEG-PCL-PDMA/mPEG-PCL-PVBA mixed micelles, but mPEG-PCL-PDMA and mPEG-PCL-PVBA were dissolved by adding THF and methanol, respectively. The micelle size was determined by DLS and the morphology was investigated by TEM.

pH-triggered changes in micelle size were monitored by DLS. Briefly, freshly prepared micelle dispersions were added to phosphate buffers (0.01 M) of different pH values (5.0, 6.5, and 7.4) and placed in a shaking bed at 37 °C at a rotation speed of 120 rpm for 24 h. The size distribution curve was measured by DLS.

### 2.5. Critical micelle concentration measurements

The CMC was determined using a fluorescence probe method with pyrene. The pyrene concentration was fixed at 6 × 10^–7^mol/l and the polymer concentration was kept in the range of 1.875 × 10^–8^ to 1.5 mg/ml. Fluorescence emissions at 375 and 386 nm were monitored using a F-4600 fluorescence spectrometer (Hitachi, Japan) by recording fluorescence spectra with an excitation wavelength of 335 nm. The CMC was estimated from the extrapolated cross-point of the fluorescence emission curves (intensity ratio I_384_/I_373_ at low and high concentration regions was considered).

### 2.6. DOX loading and release

DOX was loaded into the micelles using the membrane dialysis method. First, DOX (4 mg) was dissolved in DMSO (5 ml) under sonication for 20 min. Separately, mPEG-PCL-PDMA and mPEG-PCL-PVBA in a 1:1 molar ratio were dissolved in a mixture of THF and methanol with stirring for 5 h at room temperature. The polymer mixture was then added to the DOX solution. The resulting mixture was then added dropwise into deionized water (30 ml, pH 8.5) and stirred at room temperature for 24 h. The mixed micelle solution was then dialyzed against deionized water (pH 8.5) at room temperature in dark for 72 h. The solution in the dialysis bag (MWCO, 8,000–14,000) was then filtered through a 0.22-μm syringe filter to remove unloaded DOX. The control group DOX-loaded polymer micelles of mPEG-PCL-PDMA and mPEG-PCL-PVBA were similar to the mPEG-PCL-PDMA/mPEG-PCL-PVBA mixed micelles, but mPEG-PCL-PDMA and mPEG-PCL-PVBA were dissolved by adding THF and methanol, respectively. The morphologies of DOX-loaded mixed micelles were also investigated using TEM and their sizes were determined by DLS. Freeze-dried DOX-loaded micelles were dissolved in DMSO and the drug-loading content (DLC) of DOX was determined by measuring the DOX fluorescence (excitation wavelength, 481 nm; emission wavelength, 558 nm). The DLC was calculated using the following equation:

$$\mathrm{DLC}\;\left(\text{wt \%}\right)=\left(\frac{\text{weight of loaded drug}}{\text{total weight of loaded drug and polymer}}\right)\times 100\%$$

Drug release was studied using a dialysis method. A dialysis bag (MWCO, 8,000–14,000) filled with micellar solution (2 ml) was sealed and immersed in three buffer solutions of different pH (pH 7.4 and 6.5 PBS (0.01 M), and pH 5.0 acetate-buffered solution (0.01 M); 40 ml) and stored in a horizontal laboratory shaker with a constant temperature (37 °C) and shaking rate (120 rpm). At desired time intervals, release medium (4 ml) was removed and replenished with an equal volume of fresh medium. Each test was conducted in triplicate. The DOX concentration was determined by fluorescence spectroscopy. The cumulative release of DOX was calculated according to the following equation:

$$E_{r}=\frac{V_{e}\sum_{1}^{n-1}C_{i}+V_{0}C_{n}}{m_{\mathrm{drug}}}$$

where *E*_r_ is the cumulative release of DOX (%), *V*_e_ is the volume removed every time (ml), *C*_i_ is the concentration when the volume is removed (μg/ml), *V*_0_ is the volume of medium (ml), *m*_drug_ is the total mass of DOX contained in the release system (μg), and *n* is the number of samplings.

The article "Bicomponent polymeric micelles for pH-controlled delivery of doxorubicin" was retracted in 2024. Reasons: unreliable results or conclusions; concerns about the data.

### 2.7. In vitro toxicity evaluation

The standard MTT method was used to evaluate the toxicity of empty micelles and DOX-loaded micelles toward HepG-2, MCF-7, and normal L-02 cells. Cells were seeded into a 96-well plate (density, 5 × 10^4^ cells per well) and incubated in DMEM (100 μl) containing 10% fetal bovine serum (FBS) in a humidified incubator with 5% CO_2_ at 37 °C. After 24 h of culture, the medium was removed and conditioned media (100 μl) containing various concentrations of micelles, DOX-loaded micelles, or free DOX was added. The cells were then incubated at 37 °C for 48 h. Tests were conducted in triplicate for each concentration. Cells were treated with blank culture medium as a control. The cytotoxicity was measured using an MTT assay by recording the absorbance values at 570 nm using a microplate reader. The percentage viability of treated cells was calculated and compared with that of the untreated control cells.

### 2.8. Cellular uptake of micelles

The cellular uptake of free DOX and DOX-loaded polymer micelles was examined in HepG-2 cell lines. HepG-2 cells were seeded on the cover slips of a culture dish with a density of 7.5 × 10^4^ cells using RPMI 1640 medium supplemented with 10% FBS. After incubating for 24 h, free DOX, DOX-loaded mPEG-PCL-PDMA, mPEG-PCL-PVBA micelles, and mPEG-PCL-PDMA/mPEG-PCL-PVBA mixed micelles were added into the wells at the same DOX concentration of 10 μg/ml. After incubating at 37 °C for 12 h, the culture medium was discarded and the cells were washed three times with PBS. The cells were then fixed with 4% paraformaldehyde for 15 min and washed three times with PBS again. The cell nuclei were then stained with 4′,6-diamidino-2-phenylindole (DAPI) for 15 min. After washing with PBS four times, fluorescence images were recorded using confocal laser scanning microscopy (CLSM).

### 2.9. *In vivo* antitumor efficacy study

The animal experiment protocol was approved by the Animal Care Committee of Henan University. Female Swiss mice (5–6 weeks old, 20–25 g) were subcutaneously injected with H22 cells (1 × 10^6^ in PBS (200 μl) for each mouse) at the right armpit. When the tumor volume reached around 100 mm^3^, the mice were randomly divided into nine groups according to the body weight: (1) Saline; (2) DOX (5 mg/kg); (3) DOX (2.5 mg/kg); (4) mPEG-PCL-PDMA-DOX (5 mg/kg DOX equiv.); (5) mPEG-PCL-PDMA-DOX (2.5 mg/kg DOX equiv.); (6) mPEG-PCL-PVBA-DOX (5 mg/kg DOX equiv.); (7) mPEG-PCL-PVBA-DOX (2.5 mg/kg DOX equiv.); (8) mPEG-PCL-PDMA/mPEG-PCL-PVBA-DOX (5 mg/kg DOX equiv.); (9) mPEG-PCL-PDMA/mPEG-PCL-PVBA-DOX (2.5 mg/kg DOX equiv.). All groups were injected via the tail vein every 2 days. The tumor volume and mouse body weight were monitored daily. The tumor volume was estimated using the following equation:

$$\text{Tumor}\;\text{volume}=0.5\times {\left(\text{width}\right)}^{2}\times \left(\text{length}\right).$$

### 2.10. Histological analysis

On day 15 post-treatment, the mice were sacrificed. The tumors, heart, and liver were harvested immediately, fixed for 24 h in 4% paraformaldehyde, dehydrated, and embedded in paraffin. The embedded specimens were sectioned along the longitudinal axis of the tissues. The sections were stained with hematoxylin and eosin (H&E). Histological changes were observed under an optical microscope. Apoptotic cells in tumor cryosections were detected by terminal deoxyribonucleotidyl transferase (TdT)-mediated dUTP nick end labeling (TUNEL) assay following the manufacturer’s protocol and examined under a fluorescence microscope equipped with a green filter.

The article "Bicomponent polymeric micelles for pH-controlled delivery of doxorubicin" was retracted in 2024. Reasons: unreliable results or conclusions; concerns about the data.

### 2.11. Statistical analysis

Data are presented as means ± SD. A two-tailed Student’s *t*-test was used to study statistical differences in the data obtained and the *p* ≤ .05 value indicated a statistically significant difference.

## 3. Results and discussion

### 3.1. Characterization of amphipathic triblock copolymers

In this study, two types of amphipathic triblock copolymers were synthesized by reversible addition–fragmentation transfer (RAFT) polymerization. The synthetic procedure is shown in Figure 1.

**Figure 1.** Schematic diagram of the synthesis route of tri-block polymer mPEG-PCL-PDMA and mPEG-PCL-PVBA.

Diblock copolymer mPEG-PCL was synthesized by the ring-opening polymerization of ε-caprolactone in the presence of mPEG, whose hydroxyl end group initiated the ring-opening. The structure and composition of the synthesized mPEG-PCL diblock copolymer were determined by ^1^H NMR spectroscopy in CDCl_3_. As shown in Figure 2(A), the ^1^H NMR spectrum of the copolymer exhibited a sharp peak at 3.65 ppm, which was assigned to the methylene (CH_2_) protons of the PEG blocks, while methylene groups in PCL were demonstrated by signals at around 1.38, 1.66, 2.31, and 4.06 ppm. These results confirmed the successful synthesis of mPEG-PCL. As shown in Figure 2(B), proton peaks from the benzene ring of CTP were observed at 7.25–8.25 ppm, while peaks at 1.38, 1.76, and 2.3 ppm were assigned to PCL units. These results confirmed that polymer mPEG-PCL-CTP had been successfully synthesized. The synthesized DMA sample was also analyzed by ^1^H NMR spectroscopy, with the results shown in Supplementary Figure S1, the d_6_-DMSO solvent peak was observed as a strong signal at 2.45 ppm. The peaks at 8.78 and 8.66 ppm were assigned to catechol group protons, while those at 6.41–6.64 ppm were assigned to the DMA benzene ring. Furthermore, protons from the vinyl and methyl groups produced signals at 5.29–5.62 ppm and 1.84 ppm, respectively. The proton signal at 3.20 ppm was assigned to the amide linkage (–NH-CH_2_-CH_2_–). These results confirmed that the DMA monomer has been successfully synthesized. The ^1^H NMR spectrum of mPEG-PCL-PDMA is shown in Figure 2(C). The spectrum showed that individual mPEG-PCL and DMA were still present, while the vinyl protons of DMA at 5.29–5.62 ppm were not visible. This indicated complete consumption of the monomers and completion of the free radical polymerization process, confirming that mPEG-PCL-PDMA had been successfully synthesized. As shown in Figure 2(D), the characteristic peaks of mPEG-PCL and VBA were still present, but the vinyl protons of VBA at 5.2–6.0 ppm were not visible, indicating that mPEG-PCL-PVBA had also been successfully synthesized.

The article "Bicomponent polymeric micelles for pH-controlled delivery of doxorubicin" was retracted in 2024. Reasons: unreliable results or conclusions; concerns about the data.

**Figure 2.** ^1^H-NMR spectra of polymer (A) mPEG-PCL, (B) intermediate mPEG-PCL-CTP, (C) tri-block copolymer mPEG-PCL-PDMA, and (D) mPEG-PCL-PVBA.

Molecular weights of mPEG-PCL and mPEG-PCL-PVBA are determined by GPC. mPEG-PCL-CTP had number-average molar mass (Mn) of 9823 Da, with a polydispersity index (PDI) of 1.56. mPEG-PCL-PVBA had a Mn 14980 Da and a PDI of 1.80. But the GPC measurement of mPEG-PCL-PDMA was failed. That might be there is strong interaction between PDMA and the solid phase on GPC column. Dopamine side chains on PDMA are usually used as anchoring group to absorb onto various surfaces (Ma et al., 2019).

### 3.2. Characterization of polymeric micelles

Micellar size is an important parameter for micelles serving as drug carriers, because micelles with sizes over 200 nm are easily cleared by reticuloendothelial system (RES) *in vivo* (Baish et al., 2011; Maeda & Matsumura, 2011). The micelle particle size was characterized by DLS. As shown in Table 1, the particle size of polymeric micelles measured by DLS was less than 100 nm and the size distributions were narrow, indicating that the micelles were potential drug carriers. The TEM images showed that the self-assembly micelles were spherical in shape with diameters of <100 nm (Figure 4). Therefore, the micellar size determined by TEM correlated well with that measured by DLS. CMC determination experiments were conducted using pyrene as a fluorescent probe, as shown in Table 1. The CMCs of polymeric micelles of mPEG-PCL-PDMA, mPEG-PCL-PVBA, and mPEG-PCL-PDMA/mPEG-PCL-PVBA were 0.52, 3.7, and 0.39 mg/l, respectively. The lowest CMC value of the bicomponent micelle was originated from the complexation between two polymers through borate bonds between mPEG-PCL-PVBA and mPEG-PCL-PVBA, which could be illustrated on FTIR spectra (Supplementary Figure S2). Therefore, this kind of polymeric micelles would be more stable during dilution when entering blood circulation.

**Table 1.** Characteristics of polymer micelles.

Polymer micelles	Size (d.nm)	PDI^a^	CMC^b^ (mg/L)
mPEG-PCL-PDMA	55.29	0.157	0.52
mPEG-PCL-PVBA	47.61	0.147	3.7
mPEG-PCL-PDMA/mPEG-PCL-PVBA	65.99	0.190	0.39

a Polydispersity of micellar sizes.

b Critical micelle concentration determined using pyrene as a fluorescent probe.

The article "Bicomponent polymeric micelles for pH-controlled delivery of doxorubicin" was retracted in 2024. Reasons: unreliable results or conclusions; concerns about the data.

### 3.3. pH-triggered changes in micelle size

The pH-responsive behavior of polymeric micelles was further demonstrated by measuring the size profiles with changing pH. The changes in size of micelles with or without borate bonds in response to different pH levels are shown in Figure 3. The size distributions of polymeric mixed micelles of mPEG-PCL-PDMA/mPEG-PCL-PVBA showed obvious changes under acidic conditions (pH 5.0 and 6.5), but were stable under physiological conditions (pH 7.4). This resulted from the borate linkages breaking under acidic conditions, causing the polymer micelles containing pH-sensitive borate linkages to dissociate. In contrast, mPEG-PCL-PDMA and mPEG-PCL-PVBA micelles without borate bonds remained almost unchanged under all pH conditions. The pH-sensitive micelle DDS will remain stable and protect its payload from being cleared in blood circulation. Furthermore, when entering the acidic conditions of the tumor tissue, the loaded drug will be released to enhance the therapeutic effect.

**Figure 3.** Particle size variation of micelles under at different pH: (A) mPEG-PCL-PDMA, (B) mPEG-PCL-PVBA, and (C) mPEG-PCL-PDMA/mPEG-PCL-PVBA.

### 3.4. Drug loading and release from copolymer micelles

DOX is among the most commonly used chemotherapeutic agents clinically and is a popular model anticancer drug for fundamental studies. In this study, DOX was used as a model drug to be loaded into the polymeric micelles. The average particle size of the DOX-loaded micelles was larger than that of the blank micelles, which might be due to the larger volume of micelles after the hydrophobic micelle core was loaded with the drug. TEM images showed that the DOX-loaded micelles were spherical in shape (Figure 4). The drug-loading contents of mPEG-PCL-PDMA-DOX, mPEG-PCL-PVBA-DOX, and mPEG-PCL-PDMA/mPEG-PCL-PVBA -DOX were 10.1, 8.1, and 9.7%, respectively (Table 2). Drugs often exist in the delivery systems as hydrates, and in various crystalline and amorphous forms. These different drug forms determine the stability of the drug-loaded preparation. In general, in drug delivery, the amorphous state has a higher dissolution rate than the crystalline form, resulting in higher bioavailability. X-ray diffraction (XRD) analysis was used to study the solid forms of DOX within the formulations, as shown in Supplementary Figure S3. The results indicated that DOX in the drug-loaded preparation was embedded in the micelle in an amorphous form.

**Figure 4.** Transmission Electron Micrograph of blank and Drug-loaded micelles: (A) mPEG-PCL-PDMA, (B) mPEG-PCL-PVBA, (C) mPEG-PCL-PDMA/mPEG-PCL-PVBA and (D) mPEG-PCL-PDMA-DOX, (E) mPEG-PCL-PVBA-DOX, and (F) mPEG-PCL-PDMA/mPEG-PCL-PVBA-DOX.

The article "Bicomponent polymeric micelles for pH-controlled delivery of doxorubicin" was retracted in 2024. Reasons: unreliable results or conclusions; concerns about the data.

**Table 2.** Characteristics of DOX-loaded polymer micelles.

Polymer micelles	Size (d.nm)	PDI	DLC (%)
mPEG-PCL-PDMA-DOX	100.1	0.128	10.1
mPEG-PCL-PVBA-DOX	81.77	0.129	8.1
mPEG-PCL-PDMA/mPEG-PCL-PVBA-DOX	85.79	0.145	9.7

As a drug carrier, polymeric nanoparticles should be engineered with high stability to achieve a long circulation time and minimize premature drug release following intravenous injection (Zhong et al., 2015; Pramanik et al., 2016). As shown in Supplementary Figure S4, the nano-loaded micelles maintained relative stability when the dilution factor reached 500. Furthermore, DLS was used to investigate the aggregation behavior of DOX-loaded micelles by measuring their particle sizes after incubation with 10% FBS. As shown in Supplementary Figure S5, the average sizes of all DOX-loaded micelles did not significantly change after 48 h of incubation, indicating considerable serum stability. Furthermore, after being stored in aqueous media for one month, the size of the DOX-loaded polymeric micelles remained almost unchanged (Supplementary Figure S6). These results indicated that the drug-loaded preparation was highly stable and could be applied to a DDS.

The release profiles of DOX-loaded polymeric mixed micelles were examined *in vitro* in solution at pH 4.0, 5.0, and 7.4. As shown in Figure 5(C), the mPEG-PCL-P(DMA-b-VBA)-DOX micelles showed sustained release, with the release rates closely related to the environment pH. At pH 7.4, less than 30% of DOX was released after 72 h, indicating that mPEG-PCL-PDMA/mPEG-PCL-PVBA -DOX was relatively stable under physiological conditions. Meanwhile, significantly accelerated DOX release from mPEG-PCL-PDMA/mPEG-PCL-PVBA -DOX of 43% and 72% was observed at pH 6.5 and 5.0, respectively, within 72 h. This was attributed to the borate bond being highly sensitive to acid, with its cleavage resulting in accelerated drug release. As a control, DOX-loaded mPEG-PCL-PDMA and mPEG-PCL-PVBA polymeric micelles without borate bonds were also studied under the same conditions (Figure 5(A,B)). The DOX release profiles showed no significant differences. Under acidic environments at pH 6.5 and 5.0, drug release showed a slight pH-dependent change, which should be related to the inherent pH-sensitivity of DOX. Therefore, the mixed micelles should protect DOX from inaction during blood circulation, reaching the target tissues and rapidly releasing after cell internalization in endosomes/lysosomes with a lower pH value (Yoo et al., 2002).

**Figure 5.** The release curve of polymer drug-loaded micelle *in vitro*: (A) mPEG-PCL-PDMA-DOX, (B) mPEG-PCL-PVBA-DOX, and (C) mPEG-PCL-PDMA/mPEG-PCL-PVBA-DOX.

The article "Bicomponent polymeric micelles for pH-controlled delivery of doxorubicin" was retracted in 2024. Reasons: unreliable results or conclusions; concerns about the data.

### 3.5. Cytotoxicity of copolymer micelles

The biocompatibility of a DDS is important for practical applications. The cytotoxicity of blank polymer micelles was tested against MCF-7, HepG-2, and normal hepatocyte L-02 cells using an MTT assay. As shown in Supplementary Figure S7, the cell viability rates of all blank micelles were above 80% following 48 h of incubation, demonstrating that the blank micelles were markedly nontoxic and biocompatible up to a concentration of 400 μg/ml. To estimate the potential utility for antitumor drug delivery, MCF-7, HepG-2, and L-02 cells were employed to determine the cytotoxicity of DOX-loaded micelles, using free DOX as a positive control. The IC50 values of various DOX-loaded micelles and free DOX are summarized in Table 3. As shown in Figure 6, the cytotoxicity of the DOX-loaded micelles was dose-dependent. Free DOX appeared to show higher *in vitro* toxicity toward each cell compared with the other polymer micelles, possibly owing to the faster endocytosis process and direct transportation to the nucleus (Hu et al., 2010; Song et al., 2013). Notably, cytotoxicity assays showed that DOX-loaded polymer mixed micelles were more toxic than the other two micelle formulations. By augmenting the DOX concentration, the cytotoxicity of pH-sensitive DOX-loaded polymer mixed micelles became similar to that of free DOX. This might be due to the entry of pH-sensitive micelles through endocytosis and drug release into the cytoplasm triggered by endosome pH being quick and efficient processes (Cheng et al., 2012). Compared with free DOX, the DOX-loaded micelles exhibited significantly reduced cytotoxicity toward L-02 cells, which was probably due to the slower uptake of DOX-loaded micelles by L-02 cells. The large difference in cytotoxicity between free and formulated DOX indicated that the micellar formulations protected normal cells (Qin et al., 2017).

**Figure 6.** Viability of the activity of adriamycin micelles and adriamycin-naked drugs on (A) HepG-2, (B) MCF-7 (C), and L-02 cells (Culture with 48 h, *n* = 3).

**Table 3.** Half-inhibitory concentration (IC_50_) of DOX-loaded micelles and free DOX on HepG-2, MCF-7 and L02 cells for 48 h.

Drug preparation	IC50 (µg/mL)	
	HepG-2 cells	MCF-7 cells
mPEG-PCL-PDMA-DOX	7.840	5.364
mPEG-PCL-PVBA-DOX	8.051	5.602
mPEG-PCL-PDMA/mPEG-PCL-PVBA-DOX	5.242	2.908
Free DOX	3.495	1.958

### 3.6. Cellular uptake analysis

In the present study, various intracellular drug release behaviors of DOX⋅HCl and DOX-loaded micelles were investigated in HepG-2 cells by CLSM after incubation for 12 h. As shown in Figure 7, the pH-sensitive DOX-loaded mPEG-PCL-P(DMA-b-VBA) micelles showed relatively strong red fluorescence in the nucleus, while the DOX-loaded micelles without pH-sensitive borate ester bonds showed red fluorescence mainly in the cytoplasm and more weakly in the nuclei. This was due to the lysosomal acidic microenvironment triggering borate bond dissociation and DOX release from the micellar cores into the cells. The accumulation of DOX-loaded micelles was lower than that of free DOX with the same incubation time, probably because free DOX diffused directly through the cell membrane owing to its low molecular weight and elimination by P-glycoprotein, resulting in lowered phagocytosis (Li et al., 2014). The results showed that these biodegradable copolymer micelles could effectively release drugs into tumor cells, and that the pH-sensitive group did not reduce the cellular uptake capacity.

The article "Bicomponent polymeric micelles for pH-controlled delivery of doxorubicin" was retracted in 2024. Reasons: unreliable results or conclusions; concerns about the data.

**Figure 7.** CLSM images of HepG-2 cells following 12 h incubation with (A) mPEG-PCL-PDMA/mPEG-PCL-PVBA-DOX, (B) mPEG-PCL-PDMA-DOX, (C) mPEG-PCL-PVBA-DOX, (D) Free DOX (DOX dosage: 15 µg/mL, DOX is red fluorescence, cell nuclei stained by DAPI (blue), the scale bars correspond to 50 µm in all the images).

### 3.7. In vivo antitumor efficacy test

The *in vivo* antitumor activities of DOX-loaded micelles were assessed in mice bearing H22 tumor xenografts. Saline, free DOX, and DOX-loaded micelles were injected into the mice at the tail vein when the tumor volume was ∼100 mm^3^. Changes in tumor volume and body weight were recorded daily. As shown in Figure 8(A), tumors in the saline treatment group showed vigorous growth. In contrast, tumor growth was dramatically suppressed by treatment with various DOX formulations. The best antitumor efficiency was observed in the group treated with pH-sensitive DOX-loaded mPEG-PCL-P(DMA-b-VBA) micelles (dose, 5 mg/kg), owing to effective cellular uptake and rapid DOX release. At the end of the trial, the mean tumor volume was just 710.2 mm^3^, which was smaller than those of the other groups. Even DOX-loaded pH-insensitive micelles showed a better antitumor effect than free DOX at the same dose, which was attributed to free DOX lacking a protective vehicle, allowing it to be easily recognized and cleared by the RES. Therefore, the drug-loaded micelles showed intensive antitumor efficacy, probably owing to accumulation at the target tumor sites and accelerated release in tumor cells. Comparing the antitumor effects of different doses of the same preparation showed that the high-dose group (dose, 5 mg/kg) was more effective than the low-dose group (dose, 2.5 mg/kg), demonstrating that the antitumor effect of the preparation was concentration-dependent.

**Figure 8.** *In vivo* antitumor efficacy of the DOX-loaded micelles (*n* = 12). H22 tumor (A) growth curves and (B) body weight variation of mice after intravenous injection of different formulations of DOX. (*p < .05,**p <.01,***p < .001).

The article "Bicomponent polymeric micelles for pH-controlled delivery of doxorubicin" was retracted in 2024. Reasons: unreliable results or conclusions; concerns about the data.

Body weight change is an indicator of systemic toxicity. Therefore, changes in body weight during drug treatment were recorded. As shown in Figure 8(B), the body weight of the free DOX group (dose, 5 mg/kg) decreased gradually during treatment. This showed that free DOX was clearly toxic to mice. In contrast, mice treated with saline and DOX-loaded micelles showed a steady gain in body weight, suggesting that DOX-loaded micelles could markedly reduce the toxicity of therapeutic agents toward normal tissues and organs. These results indicated that DOX-loaded pH-sensitive micelles possessed both the most remarkable tumor inhibition efficacy and the lowest systemic toxicity, demonstrating that the pH-sensitive micelles are ideal drug delivery vehicles for DOX.

To further illustrate the improved anticancer efficacy of the pH-sensitive drug delivery micelles, H&E-stained images of the solid tumors were observed (DOX dose, 5 mg/kg). As shown in Figure 9, in the saline group, most normal tumor cells were observed, while a few necrotic regions were observed in the free DOX, mPEG-PCL-PVBA-DOX, and mPEG-PCL-PDMA-DOX groups. Notably, a larger necrosis region was observed in the mPEG-PCL-PDMA/mPEG-PCL-PVBA DOX group, as manifested by cell shrinkage, nuclei lysis, and membrane integrity destruction. These results suggested that the pH-sensitive DOX-loaded mixed micelles were a more efficient cancer therapy for inducing tumor cell necrosis and reducing tumor cell proliferation. Furthermore, the H&E-stained images of the heart and liver from the saline and DOX-loaded micelle groups showed no appreciable abnormality or noticeable organ damage. However, a large number of necrotic regions were observed in the free DOX group. This suggested that DOX-loaded micelles had good biocompatibility.

**Figure 9.** Histological assay of tumor, liver and heart sections excised from H22 tumor-bearing mice (DOX dosage: 5 mg/kg, Tumor: ×200, Heart: ×400, Liver: ×200).

TUNEL analysis was used to verify the degree of apoptosis after treatment with different DOX formulations. DNA fragments at the early stage of apoptosis were stained green using fluorescein isothiocyanate (FITC). As shown in Figure 10, the green fluorescence intensity was strongest in the pH-sensitive DOX-loaded mixed micelles group, indicating the best antitumor effect compared with the other groups. Meanwhile, almost no green fluorescence was observed in the saline group, and the free DOX group showed weak green fluorescence. The increased apoptosis of tumor cells caused by pH-sensitive DOX-loaded mixed micelle treatment further demonstrated their superiority in cancer therapy.

The article "Bicomponent polymeric micelles for pH-controlled delivery of doxorubicin" was retracted in 2024. Reasons: unreliable results or conclusions; concerns about the data.

**Figure 10.** Immunohistochemical analyses of tumor tissues from H22 tumor-bearing mice. Green: apoptotic cells, Blue: DAPI stained nucleus. (All images: ×200 magnification, DOX dosage: 5 mg/kg).

## 4. Conclusion

In this study, a two-component micelle was prepared from the mixture of phenylboronic acid-containing and catechol-containing block copolymer, which could be used in a pH responsive DDS. The pH-sensitivity of the micelle comes from the intermolecular borate ester bonds formed between the componential copolymers. *In vitro* experiments verified the pH-responsive release of DOX-loaded the bicomponent micelles, compared to the release profiles of the mono-component ones. Cytotoxicity studies showed that the pH-sensitive DOX-loaded bicomponent micelles had significantly enhanced *in vitro* cytotoxicity compared with the pH-insensitive DOX-loaded mono-component micelles, which was consistent with the confocal laser scanning microscopy results. Besides, the bicomponent micelles showed enhanced anticancer activity *in vivo*. Therefore, the bicomponent micelles are highly promising and possess obvious advantages as smart drug delivery vehicles in cancer therapy.

## Supplementary Material

Supplemental Material
